# Identification of a Necroptosis-Related Prognostic Signature and Associated Regulatory Axis in Liver Hepatocellular Carcinoma

**DOI:** 10.1155/2022/3968303

**Published:** 2022-07-09

**Authors:** Aoxiao He, Zhihao Huang, Jiakun Wang, Hongcheng Lu, Rongguiyi Zhang, Linquan Wu, Qian Feng

**Affiliations:** ^1^Department of General Surgery, Second Affiliated Hospital of Nanchang University, Nanchang, China; ^2^Department of Emergency, Second Affiliated Hospital of Nanchang University, Nanchang, China

## Abstract

**Background:**

Liver hepatocellular carcinoma (LIHC) ranks the sixth in global cancer incidence with poor prognosis. Necroptosis is a kind of regulated cell death and has been proved to be of significance in cancer occurrence and progression. However, few studies comprehensively discuss the potential applications of necroptosis-related genes (NRGs) in the prognostic evaluation and immunotherapy of LIHC.

**Methods:**

The prognostic signature in the present study was built up using LASSO Cox regression analysis. Integrated bioinformatics tools were utilized to explore the potential mRNA-miRNA-lncRNA regulatory axis in LIHC. Furthermore, qRT-PCR method was used to verify the EZH2 expression in LIHC tissues. Furthermore, prognostic performance of EZH2 in LIHC was assessed by Kaplan-Meier method.

**Results:**

A total of 14 NRGs were differentially expressed in LIHC tissues. The overall genetic mutation status of these NRGs in LIHC was also shown. NRGs were significantly correlated with programmed necrotic cell death, as well as Toll-like receptor signaling pathway in GO and KEGG pathway analysis. Kaplan-Meier analysis revealed that ALDH2, EZH2, NDRG2, PGAM5, RIPK1, and TRAF2 were related to the prognosis. A prognostic signature was constructed by these six genes and showed medium to high accuracy in the prediction of LIHC patients' prognosis. Further analysis revealed that NRGs were correlated with pathological stage, immune infiltration, and drug resistance in LIHC. Moreover, we identified a potential lncRNA TUG1/miR-26b-5p/EZH2 regulatory axis in LIHC, which might affect the progression of LIHC. qRT-PCR suggested a higher mRNA level of EZH2 in LIHC tissues. And a poor overall survival rate was detected in LIHC patients with high EZH2 expression. Moreover, EZH2 expression and cancer stage were identified as the independent risk factors affecting LIHC patients' prognosis.

**Conclusion:**

In the present study, we conducted comprehensive bioinformatic analyses and built up a necroptosis-related prognostic signature containing four genes (ALDH2, EZH2, NDRG2, and PGAM5) for patients with LIHC, and this prognostic signature showed a medium to high predictive accuracy. And our study also identified a lncRNA TUG1/miR-26b-5p/EZH2 regulatory axis, which might be of great significance in LIHC progression. In addition, based on the data from our center, the result of qRT-PCR and survival analysis showed a higher mRNA level of EZH2 in LIHC tissues and an unfavorable prognosis in high EZH2 expression group, respectively.

## 1. Introduction

Liver hepatocellular carcinoma (LIHC) ranks the sixth in global cancer incidence and has become the fourth leading cause of cancer death worldwide with 8.2% mortality rate. In 2018, LIHC causes over 700000 cancer-related deaths [1]. Over 50% LIHC patients were diagnosed at advanced stage, and the treatment options are limited, which leads to a high mortality. The lack of meaningful methods to detect LIHC and the absence of symptoms in the early stages lead to this situation [2]. Although systemic treatment, including hepatectomy, chemotherapy, targeted therapy, and immune therapy, can significantly improve patients' survival time. However, most patients face the risk of recurrence and metastasis [3]. In these circumstances, to explore the potential biomarkers for LIHC patients is of clinical significance.

Necroptosis is a novel mechanism of regulated cell death mediating by RIP1, RIP3, and MLKL [4, 5]. Some studies indicated that necroptosis was involved in the occurrence and progression of various diseases, including Parkinson disease, infectious disease, and cancer [5–7]. And there was a study indicating that necroptosis may accelerate cancer metastasis and T cell death [8] and necroptosis may activate and enhance antitumor immunity [4]. Previous studies reported that some of members in NRGs could affect LIHC patients' prognosis. For instance, depleting PGAM5 expression inhibited tumor growth and increased the 5-fluorouracil sensitivity of LIHC cells, and high PGAM5 expression was associated with an unfavorable prognosis in LIHC patients [9]. And Yao et al. suggested that LIHC patients with GG genotype in the RIPK1 rs2272990 SNP were correlated with decreased survival rate after hepatectomy [10]. The above studies indicated that NRGs might be potential biomarkers for prognosis assessment of LIHC.

Owing to the continuous updates and development of bioinformatic technique, using big data to study the molecular mechanisms of diseases and to explore biomarkers for prognosis, diagnosis, and therapy becomes feasible. At present, necroptosis-related prognostic signatures for kidney renal clear cell carcinoma, esophageal adenocarcinoma, and pancreatic adenocarcinoma have been established with high predictive accuracy [11–13]. However, as for LIHC, few studies focus on this field. Thus, in the current study, bioinformatic methods were utilized to construct a necroptosis-related prognostic signature for LIHC patients, to explore the correlations between NRGs and immune infiltration and drug sensitivity, and to seek out related regulatory axis in LIHC, which might provide novel insights in prognostic evaluation and molecular mechanisms of LIHC.

## 2. Materials and Methods

### 2.1. Datasets and Processing

On October 1st, 2021, we downloaded the RNA sequencing data and the corresponding clinical characteristics of LIHC patients from TCGA database (*n* = 371). The expression data was normalized to transcript per kilobase million (FPKM) values for the further analyses. Meanwhile, standardized copy number variation (CNV) data from TCGA-LIHC dataset was downloaded in UCSC Xena website. R software (version 4.0.5) and several online bioinformatic platforms were used to perform the analyses in the current study.

### 2.2. Expression Status, Genetic Mutation Analysis, and Functional Enrichment Analysis

By reviewing the previous literatures, we obtained 17 necroptosis-related genes which are RIPK1, RIPK3, MLKL, TLR2-4, TNFRSF1A, PGAM5, ZBP1, NR2C2, HMGB1, CXCL1, USP22, TRAF2, ALDH2, EZH2, and NDRG2 [6, 14–21]. The expression level of NRGs in LIHC tissues and normal liver tissues was visualized by “limma” and “reshape2” package in R, which was compared by Wilcoxon test. Then, we used “maftools” package to calculate the mutation frequency of necroptosis-related genes. Based on “RCircos” package, the chromosome location of NRGs and CNV alteration was presented. Using Metascape (https://metascape.org), a web portal to predict the interactions of gene set, Gene Ontology (GO) analysis and Kyoto Encyclopedia of Genes and Genomes (KEGG) analysis were performed to assess the potential biological functions and molecular mechanisms of NRGs in LIHC [22]. The threshold of GO and KEGG pathway analysis was set as a *p* value of 0.01, a minimal overlap of 3, and a minimal enrichment of 1.5.

### 2.3. Prognosis Analysis and Construction of Necroptosis-Related Prognostic Signature

Kaplan-Meier methods were performed to identify the prognostic NRGs, and log-rank test was applied to calculate the *p* values, hazard ratio (HR), and 95% confidence interval (CI). Based on prognostic NRGs, a prognostic signature was built up using LASSO Cox regression model. Riskscore = ∑_*i*=1_^*n*^(Expi × Coei). Setting the median risk score as the cutoff, patients were divided into low- and high-risk groups. OS curves of the two groups were compared by Kaplan-Meier analysis, and the predictive accuracy of the prognostic model was assessed by time ROC curve. In addition, Spearman's correlation analysis was used to explore the relationship between risk score and infiltrating level of immune cells in LIHC tissues.

### 2.4. Stage Plots, Immune Infiltration Analysis, and Drug Sensitivity Analysis of NRGs Associated with Risk Score

The correlation between pathological stage and the expression level of ALDH2, EZH2, NDRG2 and PGAM5 in LIHC tissues was visualized by violin plots. Next, TIMER (https://cistrome.shinyapps.io/timer) was used to illustrate the association between immune cell infiltration and the expression of NRGs associated with risk score. And the comparison of infiltration levels among LIHC tissues with different somatic copy number alterations (SCNAs) for NRGs associated with risk score were also visualized. Moreover, Pearson's correlation analysis was conducted to show the correlation between NRGs associated with risk score and drug sensitivity data from Genomics of Drug Sensitivity in Cancer (GDSC).

### 2.5. mRNA-miRNA-lncRNA Network Construction

The miRNA targets of NRGs associated with risk score were detected in TargetScan (http://www.targetscan.org/), miRDB (http://mirdb.org/), and StarBase (http://starbase.sysu.edu.cn/), respectively. The expression level and prognostic performance of the miRNA targets which were included in the intersection among these three databases were shown. According to the above miRNA targets, upstream lncRNA targets binding to miRNAs were explored by StarBase (http://starbase.sysu.edu.cn/) and LncBase (https://carolina.imis.athena-innovation.gr/). Similarly, the most promising lncRNA targets were detected with Student's *t*-test by TCGA-LIHC dataset.

### 2.6. Validation of the Expression Level and Prognosis Performance of EZH2 in LIHC

Forty LIHC tissues and corresponding normal liver tissues from patients without any treatment preoperatively were collected. The expression of EZH2 in LIHC tissues and normal liver tissues was compared by Student's *t*-test. Kaplan-Meier method was conducted to compare the prognosis between high- and low-EZH2 expression groups. Moreover, taking the clinical characteristics and EZH2 expression into consideration, univariate and multivariate Cox regression analyses were conducted to identify the independent risk factors affecting patients' prognosis. The above plots were drawn by GraphPad Prism7 software (GraphPad, Inc., La Jolla, CA, USA). In addition, the study was approved by the Ethics Committee of the Second Affiliated Hospital of Nanchang University, and each patient provided written informed consent.

## 3. Results

### 3.1. The Expression and Genetic Mutation Landscape of NRGs in LIHC

The mRNA levels of all 17 NRGs in LIHC tissues and normal liver tissues were visualized in Figure 1(a). Compared with normal liver tissues, the expression levels of RIPK1, MLKL, PGAM5, NR2C2, HMGB1, USP22, TRAF2, and EZH2 were increased while the expression levels of TLR3, TLR2, TLR4, TNFRSF1A, ALDH2, and NDRG2 were decreased in LIHC tissues (all *p* < 0.05).  Figure 1(b) showed the simple nucleotide variations (SNVs) of NRGs in TCGA-LIHC dataset, and a total of 92% (23/25) LIHC samples were presented with genetic mutations. Of these NRGs, USP22 was the gene with the highest frequency of mutation. And we found that missense was the only type of variant classification, and *C*>T was the most common SNV class (Figure 1(c)). The results of CNV analysis were shown in Figure 1(d), which indicated that RIPK1, NDRG2, EZH2, TRAF2, USP22, NR2C2, TNFRSF1A, and TLR2 showed CNV amplification while the others showed widespread CNV deletion. The location of NRGs on chromosomes was showed in Figure 1(e).

### 3.2. GO and KEGG Analyses of NRGs in LIHC

GO and KEGG pathway analyses were performed to predict the potential biological functions and molecular mechanisms of these 17 NRGs and confirm whether they were associated with necroptosis in LIHC. In Figures 2(a) and 2(b), these NRGs were primarily correlated with programmed necrotic cell death, positive regulation of interleukin-8 production, I-kappaB phosphorylation, I-kappaB kinase/NF-kappaB signaling, and cytokine binding in GO analysis. And corresponding protein-protein interaction (PPI) network was visualized in Figure 2(b). The PPI network of KEGG pathway analysis was shown in Figure 2(c). KEGG pathway analysis indicated these genes were associated with TNF signaling pathway, NF-kappa B signaling pathway, Toll-like receptor signaling pathway, and Herpes simplex infection (Figure 2(d)).

### 3.3. Construction of a Necroptosis-Related Prognostic Signature

Kaplan-Meier survival curves revealed that LIHC patients with high EZH2, PGAM5, RIPK1, and TRAF2 expression showed an unfavorable OS rate, while patients with high ALDH2 and NDRG2 expression were associated with a better OS rate (Figure 3). Next, a LASSO Cox regression prognostic model was constructed by these 6 prognostic NRGs. Riskscore = (−0.1139)∗ALDH2 + (0.247)∗EZH2 + (−0.0678)∗NDRG2 + (0.1848)∗PGAM5. The coefficient and partial likelihood deviance were revealed in Figures 4(a) and 4(b), respectively. According to the median risk score, patients were grouped into low- and high-risk group.  Figure 4(c) showed the distribution of risk score, survival status, and the expression levels of NRGs in TCGA-LIHC dataset. The patients were listed from low- to high-risk score. On the whole, LIHC patients with high EZH2 expression, high PGAM5 expression, low NDRG2 expression, and low ALDH2 expression tended to have a high risk score, thus leading to a relatively poor prognosis. As was expected, LIHC patients in high-risk group showed a worse OS rate than low-risk group (Figure 4(d), *p* = 0.0000147, 2.6 years vs. 6.7 years). Area under the curve (AUC) of 1-year, 3-year, and 5-year ROC curve was 0.743, 0.684, and 0.678, respectively (Figure 4(e)). The relationship between risk score and immune infiltrating level in LIHC tissues was also analyzed. As shown in Figure 5, risk score had a closely positively relationship with the expression of B cell (Figure 5(a), *p* = 4.55*e* − 14, Cor = 0.38), CD4+ T cell (Figure 5(b), *p* = 4.71*e* − 15, Cor = 0.39), neutrophil (Figure 5(d), *p* = 1.1*e* − 14, Cor = 0.39), macrophage (Figure 5(e), *p* = 1.41*e* − 11, Cor = 0.34), and myeloid dendritic cell (Figure 5(f), *p* = 7.76*e* − 17, Cor = 0.40).

### 3.4. Necroptosis-Related Genes Correlated with Pathological Stage, Immune Infiltration, and Drug Resistance in LIHC

In Figure 6(a), it showed that the expression of ALDH2 (*p* = 0.000302) and NDRG2 (*p* = 0.0321) decreased as the pathological stage increased. However, the expression of EZH2 increased as the pathological stage increase. We then selected EZH2, ALDH2, and NDRG2 to explore their relationship with immune infiltration in LIHC, respectively. The result showed that a positive correlation existed between EZH2 and the immune abundance of B cells (*p* = 1.24*e* − 20, cor = 0.474), CD8+ T cells (*p* = 9.30*e* − 08, cor = 0.284), CD4+ T cells (*p* = 3.84*e* − 13, cor = 0.378), macrophage (*p* = 3.22*e* − 17, cor = 0.436), neutrophils (*p* = 7.02*e* − 13, cor = 0.374), and dendritic cells (*p* = 1.38*e* − 18, cor = 0.453). ALDH2 expression showed negative correlation with B cell (*p* = 6.25*e* − 06, cor = −0.241), CD8+ T cell (*p* = 1.13*e* − 04, cor = −0.207), CD4+ T cell (*p* = 1.60*e* − 05, cor = −0.23), macrophage(*p* = 2.75*e* − 09, cor = −0.315), neutrophils (*p* = 4.85*e* − 03, cor = −0.151), and dendritic cells (*p* = 3.59*e* − 06, cor = −0.248). There was a negative association between infiltration level of B cell (*p* = 1.44*e* − 02, cor = −0.132) and NDRG2 expression in LIHC tissues (Figure 6(b)). We then found that certain SCNAs of the three prognostic NRGs could inhibit immune infiltration in LIHC (Figure 6(c)). Moreover, we evaluated the correlation between the expression of these 3 NRGs and existed drug targets to measure cancer immunotherapy target. As the results shown in Figure 6(d), drug sensitivity analysis revealed that high expression of ALDH2 was correlated with GDSC drug sensitivity, while the expression of EZH2 showed negative correlation with GDSC, and the correlation between the expression of NDRG2 with the most existed drug targets was not very significant, suggesting that EZH2 and ALDH2 may work as the potential biomarkers for drug scanning.

### 3.5. Construction of a mRNA-miRNA-lncRNA Network

Previous studies had clearly reported the function of ALDH2 in the occurrence and progression of LIHC [23]. Thus, we constructed a mRNA-miRNA-lncRNA network to find out the potential regulatory axis of EZH2 in LIHC. By searching the genomic data in miRDB, TargetScan, and StarBase, four potential miRNAs were identified, including hsa-miR-4465, hsa-miR-26a-5p, hsa-miR-26b-5p, and hsa-miR-1297 (Figure 7(a)), and the expression of hsa-miR-26a-5p and hsa-miR-26b-5p was significantly decreased in LIHC tissues (Figures 7(b) and 7(c)). Survival analysis revealed that high hsa-miR-26b-5p expression was associated with an unfavorable OS rate in LIHC patients (Figure 7(d), *p* = 0.045). Therefore, we selected hsa-miR-26b-5p as the most promising miRNA target of EZH2. The upstream lncRNAs binding to hsa-miR-26b-5p were excavated by LncBase and StarBase. The results advised TUG1, KCNQ1OT1, and GAS5 as the lncRNAs targets (Figure 7(e)). Moreover, it showed that TUG1, KCNQ1OT1, and GAS5 were elevated in LIHC tissues (Figure 7(f), *p* < 0.0001). Survival analysis suggested high TUG1 expression was linked with unfavorable OS rate in LIHC patients (Figure 7(g), *p* = 0.026). Therefore, the potential mRNA-miRNA-lncRNA regulatory axis, lncRNA TUG1/miR-26b-5p/EZH2 regulatory axis, was detected, which might influence the development of LIHC.

### 3.6. Validation of the Expression and Prognostic Value of EZH2 in LIHC

The mRNA level of EZH2 in LIHC tissues and normal liver tissues was analyzed by qRT-PCR, which showed a significant upregulation in LIHC tissues (*p* < 0.0001, Figure 8(a)). The survival data of these 40 patients were also collected, which showed a worse OS rate in high EZH2 expression group (Figure 8(b), *p* = 0.038). Univariate and multivariate Cox regression analyses suggested that EZH2 expression and nodal metastasis status, cancer stage, gender, and age were the independent risk factors affecting LIHC patients' prognosis (Figures 8(c) and 8(d), all *p* < 0.05).

## 4. Discussion

Previous studies had demonstrated that necroptosis was related to tumor cell migration and invasion regulation in many human cancer types [24]. And, necroptosis, as a form of programmed cell death, was considered as a promising approach to eliminate cancer cells [25]. The potential molecular mechanisms of NRGs and their prognostic value in LIHC were rarely discussed [26]. Elucidating the prognostic performance and potential regulatory axis of NRGs in LIHC will help clinicians to explore the effect of necrotosis on the prognosis and treatment of LIHC.

First, the mRNA levels of the 17 NRGs in LIHC tissues and normal liver tissues were visualized. The upregulated genes (RIPK1, MLKL, PGAM5, NR2C2, HMGB1, USP22, TRAF2, and EZH2) and the downregulated genes (TLR3, TLR2, TLR4, TNFRSF1A, ALDH2, and NDRG2) were selected out for further analyses. Functional enrichment analysis was conducted to confirm whether these differentially expressed NRGs had associations with necroptosis in LIHC, which showed these NRGs were correlated with programmed necrotic cell death, positive regulation of interleukin-8 production, TNF signaling pathway, NF-kappa B signaling pathway, Toll-like receptor signaling pathway, and Herpes simplex infection. The above pathways had correlations with necroptosis and tumor progression, which was proven in previous studies. And NF-kappa B signaling pathway regulated the process of inflammation and cancer progression [27]. TNF signaling pathway was of great importance in mammalian immunity and cellular homeostasis [28]. Furthermore, TNF signaling pathway was found to regulate the balance between cell survival and necroptosis [29].

In our study, survival analysis suggested that high EZH2, PGAM5, RIPK1, and TRAF2 expressions were related to an unfavorable prognosis in LIHC patients, while high ALDH2 and NDRG2 expressions were linked with a better prognosis. For better predicting LIHC patients' prognosis, the expression profile of these 6 prognostic genes in TCGA-LIHC dataset was used to build up a prognostic signature. Of these 6 genes, only EZH2, ALDH2, NDRG2, and PGAM5 were associated with risk score. In general, our prognostic signature obtained medium to high accuracy in the prediction of LIHC patients' prognosis. Previous studies had reported EZH2 was related to the progression, invasion, and metastasis of the hepatocellular carcinoma [30–32]. However, our study firstly built up a necroptosis-related prognostic signature in LIHC, which provided another biomarker for LIHC patients.

Another significant finding of the current study was that NRGs were significantly correlated with pathological stage, immune infiltration, and drug resistance in LIHC. ALDH2 decreased as the pathological stage increased, indicating that ALDH2 may serve as a tumor suppressor and inhibit LIHC progression. Hou et al. also revealed that ALDH2 opposes hepatocellular carcinoma progression by regulating AMP-activated protein kinase signaling in mice [23]. In our study, the data suggested a positive correlation between EZH2 and the immune abundance of B cells, CD8+ T cells, CD4+ T cells, macrophage, neutrophils, and dendritic cells. Interestingly, previous study had found that EZH2 is correlated with immunosuppression and poor survival in LIHC [33]. Moreover, EZH2 could inhibit PD-L1 expression in LIHC [34]. Another study found that EZH2 could suppress NK cell-mediated antitumor immunity via inhibiting CXCL10 expression in a HDAC10-dependent manner [35]. These evidences demonstrated that EZH2 may play a vital role in the antitumor immunity of LIHC.

Through mRNA-miRNA-lncRNA network, lncRNA TUG1/miR-26b-5p/EZH2 regulatory axis was identified, which might participate in the occurrence and progression of LIHC. Previous study had reported the expression level of TUG1 was increased in LIHC tissues and the expression of TUG1 promoted LIHC cell proliferation in mouse model [36]. In LIHC tissues, Wang et al. [37] indicated that miR-26b-5p decreased significantly, and it was a negative regulator of proliferation, angiogenesis, and apoptosis. Furthermore, Zhai et al. [38] found that EZH2 was significantly elevated in LIHC tissues, and high EZH2 expression showed a worse prognosis in LIHC patients. In the previous studies, EZH2 was also related to the occurrence and development of LIHC, which promoted viral carcinogenesis in patients with HBV infection [39]. The above evidences supported the findings of this study. However, more fundamental studies are urgently needed to validate this regulatory axis.

## 5. Conclusion

The major findings of the present study were as follow: first, we utilized TCGA-LIHC dataset and bioinformatic methods to construct a necroptosis-related prognostic signature containing four genes (ALDH2, EZH2, NDRG2, and PGAM5), which obtained medium to high predictive accuracy. Second, the current study used ceRNA network to identify a lncRNA TUG1/miR-26b-5p/EZH2 regulatory axis, which might influence the progression of LIHC. In addition, we used the data from our center to perform qRT-PCR and survival analysis, which indicated a higher mRNA level of EZH2 in LIHC tissues and an unfavorable prognosis in high EZH2 expression group, respectively. However, further in vivo and in vitro studies should be conducted to verify these results.

## Figures and Tables

**Figure 1:** Expression and genetic variation Landscape of necroptosis-related genes in LIHC. (a) The mRNA level of 17 necroptosis-related genes in LIHC. (b, c) The mutation frequency and classification of 17 necroptosis-related genes in LIHC. (d) The CNV frequency of 17 necroptosis-related genes in LIHC. The height of the column represented the alteration frequency. (e) The location on chromosomes of CNV of 17 necroptosis-related genes. Note: ∗∗*p* < 0.01, and ∗∗∗*p* < 0.001.

**Figure 2:** The enriched items in functional analysis. (a, b) The enriched items in gene ontology analysis. (c, d) The enriched items in Kyoto Encyclopedia of Genes and Genomes analysis.

**Figure 3:** Prognostic analysis of the necroptosis-related genes. Overall survival curve in LIHC patients with high/low expression of ALDH2, EZH2, NDRG2, PGAM5, RIPK1, and TRAF2.

**Figure 4:** Construction of a necroptosis-related prognostic gene signature. (a, b) The coefficient and partial likelihood deviance of prognostic signature. (c) Risk score distribution, survival status of patients, and gene expression in prognostic signature. (d, e) Overall survival curve in high/low-risk group and the ROC curve evaluating prognosis predicting performance of LIHC patients.

**Figure 5:** Riskscore correlated with immune infiltration in LIHC. The correlation between risk score and the expression of B cells (a), CD4+ T cells (b), CD8+ T cells (c), neutrophils (d), macrophage (e), and dendritic cells (f).

**Figure 6:** Necroptosis-related genes correlated with pathological stage, immune infiltration, and drug resistance in LIHC. (a) The correlation between pathological stage and ALDH2, EZH2, NDRG2, and PGAM5. (b) The correlation between immune cell infiltration and EZH2/ALDH2/NDRG2 in LIHC. (c) The correlation between copy number alteration of EZH2/ALDH2/NDRG2 and immune cell infiltration in LIHC. (d) The correlation between TLR2/NDRG2 expression and GDSC drug sensitivity. GDSC: Genomics of drug sensitivity in cancer. Note: ∗*p* < 0.05, ∗∗*p* < 0.01, and ∗∗∗*p* < 0.001.

**Figure 7:** Construction of lncRNA-miRNA-mRNA regulatory axis. (a) miRNA target of EZH2 predicted by miRDB, TargetScan, and Starbase. The expression of miR-26b-5p (b) and miR-26b-5p (c) in LIHC. (d) Overall survival curve in LIHC patients with high/low miR-26a-5p and miR-26b-5p expression. (e) lncRNA targets of miR-26b-5p predicted by LncBase and StarBase. (f) The expression of lncRNA TUG1, KCNQ1OT1, and GAS5 in LUAD. (g) Overall survival curve in LIHC patients with high and low TUG1 expression. Note: ∗∗∗*p* < 0.001, and ∗∗∗∗*p* < 0.0001.

**Figure 8:** The expression and prognosis value of EZH2 in LIHC. (a) The relative expression of EZH2 in LIHC tissues and normal tissues. (b) Survival curve revealed the overall survival of LIHC patients with high/low EZH2 expression. (c, d) Univariate and multivariate Cox regression analysis of EZH2 and clinical characters in LIHC. Note: ∗∗∗∗*p* < 0.0001.

## Data Availability

The datasets used or analyzed in this study are available from the corresponding author on reasonable request.
